The article "A Systematic Review and Meta-Analysis Comparing the Safety and Efficacy of Spinal Anesthesia and Spinal Anesthesia Combined with Obturator Nerve Block in Transurethral Resection of Bladder Tumors" was published in 2022. Journal: Emerg Med Int.

# A Systematic Review and Meta-Analysis Comparing the Safety and Efficacy of Spinal Anesthesia and Spinal Anesthesia Combined with Obturator Nerve Block in Transurethral Resection of Bladder Tumors

**DOI:** 10.1155/2022/8490462

**Published:** 2022-06-29

**Authors:** Wanxin Deng, Qiang Zhang, Hongmei Yao

**Affiliations:** Department of Anesthesiology, The First People's Hospital of Longquanyi District, Chengdu, Sichuan 610100, China

## Abstract

**Background:**

Transurethral resection of bladder tumors (TURBT) is the main surgical treatment for bladder cancer, but during TURBT, it is easy to stimulate the obturator nerve passing close to the lateral side of the bladder wall and induce involuntary contraction of the adductor muscle group of the thigh innervated by it, which will affect the surgical process and lead to adverse reactions. Obturator nerve block (ONB) helps to prevent the obturator nerve reflex. This study systematically evaluated and meta-analyzed the reports on the co-application of ONB and spinal anesthesia (SA) in TURBT in recent years to provide evidence for clinical diagnosis and treatment.

**Methods:**

The clinical randomized controlled literature studies of ONB combined with SA in TURBT published in PubMed, EMBASE, the Cochrane Library, CNKI (China National Knowledge Infrastructure), and Wanfang databases from January 2000 to December 2021 were searched. After screening the qualified literature studies, the literature quality was assessed by the Jadad scale. The incidence of obturator nerve reflex, the incidence of bladder perforation, length of hospital stay, and tumor recurrence rate were used as outcome indicators. The meta-analysis was performed with the *R* language toolkit.

**Results:**

A total of 444 articles were initially retrieved, and after the screening, a total of 8 articles were included in the selection, and a total of 635 patients with ureterovesical tumor resection were included. The meta-analysis showed that the use of SA + ONB anesthesia during TURBT was associated with a smaller incidence of bladder perforation (*RR* = 0.24, 95% CI (0.11, 0.53), *Z* = −3.48, *P*=0.0005), a smaller incidence of obturator nerve reflex (*RR* = 0.22, 95% CI (0.13, 0.36), *Z* = −6.11, *P*=0.0001), a significantly shorter length of hospital stay (*MD* = −1.81, 95% CI (−2.65, −0.97), *Z* = −4.24, *P*=0.0001), and a significantly lower tumor recurrence rate (*RR* = 0.46, 95% CI (0.29, 0.73), *Z* = −3.30, *P*=0.001) compared with SA alone.

**Conclusion:**

The application of SA combined with ONB in TURBT can effectively reduce the incidence of obturator nerve reflex, reduce the incidence of bladder perforation, shorten the hospital stay and reduce the tumor recurrence rate.

## 1. Introduction

Bladder cancer is a primary malignant tumor in the bladder mucosa and is one of the most common tumors of the human genitourinary system [1]. Its etiology is still not clear and may be related to genetic factors and environmental factors, and frequent urination, urgency, urinary pain, and dysuria are the main symptoms. Most patients can be seen with painless hematuria [2]. Bladder cancer mostly occurs in middle-aged and elderly people over 50 years old, and the incidence rate increases with age. The occurrence of bladder cancer is closely related to the three factors of diet, smoking, and drinking water. Therefore, the prevention of bladder cancer should also start from the source. For early noninvasive bladder cancer, transurethral resection of bladder tumors (TURBT) is the main surgical treatment [3].

However, during TURBT, the obturator nerve passing immediately lateral to the bladder wall is easily stimulated to induce involuntary contraction of the adductor muscle group of the thigh innervated, which will affect the surgical process and may lead to the occurrence of adverse effects such as incomplete tumor resection, bladder perforation, or bleeding [4, 5]. The incidence of obturator nerve reflex in unipolar bladder tumors is as high as more than 55% [6]. General anesthesia is a traditional method to prevent obturator nerve reflex, but it is not suitable for elderly patients; epidural local anesthesia and spinal anesthesia are commonly used spinal anesthesia (SA) methods, which can inhibit the contraction of adductor muscle conducted by sensory fibers, but do not completely block obturator nerve reflex [7]. Obturator nerve block (ONB) is performed by an ultrasound-guided puncture to locate the obturator nerve and perform local anesthesia so as to reduce obturator nerve emission [8].

In the study by Krishan et al. [9], 8 articles were included for meta-analysis, but this study included a retrospective analysis, and the quality of evidence was low. Therefore, in our study, a meta-analysis was performed again by including randomized controlled trials to further clarify the effectiveness of ONB-assisted in TURBT in order to provide a reference for clinical practice.

## 2. Materials and Methods

### 2.1. Inclusion Criteria

①Study types: all the included studies were randomized controlled trials (RCTs), and the languages of literature studies were Chinese and English. Given the rigor of the procedure, we excluded observational studies with two contrast cohorts; studies of review nature, conference proceedings, expert consensus, case series, and case studies would also be excluded; ②Study subjects: all patients underwent TURBT. Before the operation, all patients were diagnosed with bladder tumor by computed tomography, B ultrasound, or cystoscopy; the tumor was located in the lateral bladder wall. We did not limit the location of the tumor to unilateral or unilateral, but the tumor was located in the area innervated by the obturator nerve; experimental studies with animals were excluded. ③Intervention measures: all studies were carried out in a randomized controlled group. Spinal anesthesia was used before surgery in both groups. The unlimited anesthesia method was an arachnoid injection, epidural injection, or a combination of the two. In the experimental group, after the completion of spinal anesthesia, the obturator nerve block was performed, the inguinal approach or pubic approach was selected, needle puncture was performed with ultrasound imaging, and local anesthetic drugs were injected for obturator nerve block, or the obturator nerve was located using a nerve stimulator under ultrasound and the local anesthetic block was given. ④Outcome indicators: efficacy indicators. We used the incidence of cystocentesis and the incidence of obturator nerve reflex as short-term efficacy and safety indicators, and the length of hospital stay and tumor recurrence rate as long-term efficacy indicators.

### 2.2. Literature Search

①Search strategy: a search strategy (“obturator nerve block”|“ONB”) AND (“transurethral resection of bladder tumors”| TURBT). Perform a wide range of keyword search. ②Database: search PubMed, EMBASE, the Cochrane Library, CNKI (China National Knowledge Infrastructure), Wanfang database. ③Filter setting: we perform a computer search for the database with filter set in the search website, set the literature publication time (January 2000–December 2021), and the literature type (Only RCTs).

### 2.3. Selection of Literature Studies

After two researchers independently completed the search, the literature data were entered into EndNote X9 software for subsequent management. Duplicate files were removed by using the de-duplication function of the software. Two researchers performed manual de-duplication of the remaining literature studies again. If the first author, study site, intervention method, and number of groups were all the same, it could be considered that two literature studies were duplicated, and only one of them was retained. After de-duplication, two researchers read the title, abstract, and full text of the literature studies again, and excluded the unqualified literature studies. In case of any dispute in the process, a third person can intervene and coordinate after discussion.

### 2.4. Data Extraction and Conversion

After the screening of the literature studies, two researchers extracted the following data from the included literature studies: literature characteristics information (author, publication time, and study site), study object information (gender, age, and weight), intervention measure information (number of patients in groups, intervention method), and outcome information (outcome indicator). In order to facilitate subsequent meta-analysis, some data are converted, such as length of hospital stay, and some studies are converted to “*d*” in “*h*.”

### 2.5. Risk Assessment of Literature Bias

The risk of bias of literature studies was evaluated by the Cochrane Handbook for Systematic Reviews of Intervention provided by the Cochrane Collaboration. The following 6 aspects of literature studies were evaluated: (1) randomization method; (2) blind method; (3) implementation of allocation concealment; (4) data integrity; (5) selective reporting bias; (6) other biases, which were evaluated as “low risk,” “unclear,” and “high risk.” The Jadad score scale was used to assess the quality of the literature, with a maximum score of 5 and a score of more than 3 as excellent quality.

### 2.6. Statistical Methods

①The R Version 4.1.2, released by the *R* foundation for statistical computing, was used for analysis; ②continuous indicators were reported using mean variance (MD) effect size and 95% CI, and discrete indicators (dichotomization) were reported using the risk ratio (*RR*) effect size and 95% CI, with *P* < 0.05 indicating statistical significance; ③each primary outcome indicator was analyzed; ④forest plot was used to display the effect size; ⑤*I*^2^ analysis and *Q* were used to verify the heterogeneity of the literature, with *I*^2^ >50% or *P* < 0.1 indicating the presence of heterogeneity, random effect model was used, otherwise a fixed effect was used. The Mantel-Haenszel model was used for OR effect size, and an inverse variance model was used for SMD effect size; ⑥if it is suggested that there is heterogeneity in the literature studies, investigate the source of heterogeneity and only make a descriptive analysis when it is impossible to judge the source of heterogeneity; Subgroup analysis was performed; ⑦sensitivity analysis was performed by eliminating the results from the literature one by one; and ⑧funnel plot was used to represent the publication bias.

## 3. Results

### 3.1. Literature Screening Process and Results

Literature selection flow chart is shown in Figure 1; 444 literature studies were initially searched. After screening, a total of 8 literature studies were included in the selection, including 635 patients who underwent urethrovesical tumor resection, including 6 English literature studies and 2 Chinese literature studies.

### 3.2. Basic Characteristics of Literature Studies

The basic characteristics and intervention measures, outcome indicators, and the Jadad score of the included articles are shown in Table 1, including 5 articles using the ONB inguinal approach, 3 articles using the pubic approach, 6 articles using ONB nerve electrical stimulation, and 2 articles using only ultrasound guidance.

### 3.3. Literature Bias Assessment

In this study, all the literature studies were RCT studies, which indicated the use of the randomization method, so there was no selection bias caused by the randomization method; however, the literature studies [14, 16, 17] did not indicate the allocation concealment, and the literature studies [16, 17] did not describe the blind method, which may cause the implementation bias. The literature studies [16, 17] also did not record the data dropout cases in detail, which may cause part of the attribution bias; there was no selective reporting or other bias, as shown in Table 2.

### 3.4. Meta-Analysis Results

#### 3.4.1. Incidence of Bladder Perforation

All literature studies [10, 12, 14, 16, 17] reported an incidence of bladder perforation after SA + ONB and SA alone surgery, 238 patients were included in the SA + ONB group and 239 patients were included in the SA alone group, with no statistical heterogeneity in the literature studies (*I*^2^ = 0%, *P*=0.95). Fixed effect model analysis was used, resulting in a pooled value (*RR* = 0.24, 95% CI (0.11, 0.53), that means the incidence of bladder perforation using SA + ONB during surgery was significantly less than that using SA alone (*Z* = −3.48, *P*=0.0005). The patients were further divided into two subgroups according to the approach of ONB: the inguinal approach group and the pubic approach group. There was no statistical heterogeneity between the internal literature studies, as shown in Figure 2.

#### 3.4.2. Incidence of Obturator Reflex

In the literature studies [10, 12, 14–16], the incidence of obturator reflex after SA + ONB and SA surgery was reported, 203 patients were included in the SA + ONB group and 206 patients were included in the SA alone group. There was no statistical heterogeneity in the literature studies (*I*^2^ = 0%, *P*=0.70). The fixed effect model analysis was used to obtain the pooled value (*RR* = 0.22, 95% CI (0.13, 0.36), that means the incidence of obturator reflex using SA + ONB during surgery was significantly less than that using SA alone (*Z* = −6.11, *P* < 0.0001). The patients were further divided into two subgroups according to the approach of ONB: the inguinal approach group and the pubic approach group. There was no statistical heterogeneity between the internal literature studies, as shown in Figure 3.

#### 3.4.3. Length of Hospital Stay (d)

The literature studies [10, 16, 17] reported the length of hospital stay after SA + ONB and SA alone surgery, the unit is days (*d*), 156 patients were included in the SA + ONB group and 155 patients were included in the SA alone group, with statistical heterogeneity in the literature studies (*I*^2^ = 71%, *P*=0.03). Random effects model analysis was used to obtain the pooled value (*MD* = −1.81, 95% CI (−2.65, −0.97), that means the length of hospital stay using SA + ONB during surgery was significantly less than that using SA (*Z* = −4.24, *P* < 0.0001), as shown in Figure 4.

#### 3.4.4. The Tumor Recurrence Rate during Follow-Up Period

It has been reported in the literature studies [10, 11, 14, 17] in both SA + ONB and SA alone groups. 190 patients were included in the SA + ONB group and 195 patients were included in the SA alone group. There was no statistical heterogeneity in the literature studies (*I*^2^ = 0%, *P*=0.92). The fixed effect model analysis was used to obtain the pooled value (*RR* = 0.46, 95% CI (0.29, 0.73), that means the tumor recurrence rate using SA + ONB during surgery was significantly less than that using SA alone (*Z* = −3.30, *P*=0.001), as shown in Figure 5.

#### 3.4.5. Heterogeneity Investigation and Sensitivity Analysis

In the meta-analysis of the incidence of bladder perforation and the incidence of obturator nerve reflex, there was no statistically significant heterogeneity in the literature studies. We tried to analyze the literature studies according to different surgical approaches, but there was still no statistically significant heterogeneity within the literature studies. We performed a sensitivity analysis using impact factors for the incidence of bladder perforation, and after sequentially excluding each study, the pooled effect size of the remaining studies did not change significantly, suggesting that the results were stable as shown in Figure 6.

#### 3.4.6. Publication Bias Analysis

In the analysis of the incidence indicator of bladder perforation, all the 5 included literature studies were within the funnel, but the left and right sides were not evenly distributed, suggesting that there was a small publication bias, as shown in Figure 7.

## 4. Discussion

Anatomically, the obturator nerve arises from the anterior thigh of the anterior branch of *L*2–*L*4 and enters the minor pelvis after the medial border of the psoas muscle comes out; it progresses along the lateral wall of the minor pelvis and protrudes from the obturator canal from the minor pelvis to the thigh, dividing the anterior and posterior branches, and enters the thigh adductor muscle group through the anterior and posterior adductor brevis muscles; during the course of the obturator nerve, it abuts the bladder neck, lateral bladder wall, and prostatic urethra [18]. Therefore, when TURBT is performed in patients with lateral bladder wall tumors, obturator nerve reflexes often occur due to induced current stimulating the adjacent obturator nerve, which causes involuntary spasms or even sudden and intense movement of the thigh adductor muscle, resulting in bladder perforation, massive hemorrhage, abdominal organ injury, and extravesical spread of the tumor [19]. In previous practice, general anesthesia was applied to control the obturator nerve reflex, but general anesthesia could not be applied to older patients. Therefore, spinal anesthesia has been more widely used in TURBT, but spinal anesthesia cannot completely prevent the obturator nerve reflex [20]. Muscle relaxants are another method to control the obturator nerve reflex, but the timing, dosing interval, and dose of muscle relaxant are not well controlled [21]. Obturator nerve block, which is found to help prevent obturator nerve reflex, has received increasing attention and become another option [22].

In this meta-analysis, a total of 8 controlled clinical studies published in recent years were retrieved, with 635 patients undergoing TURBT. The results showed that the use of SA combined with ONB anesthesia could effectively reduce the incidence of obturator nerve reflex, reduce the incidence of bladder perforation, shorten the length of hospital stay, and reduce the tumor recurrence rate, which revealed that SA combined with ONB had more advantages than SA anesthesia alone. Ultrasound-guided obturator nerve block can reduce intraoperative obturator nerve reflex, make the operation more calm and accurate, do not have to worry about obturator nerve reflex and reduce the extent and depth of resection and electrocautery, which is also conducive to reducing intraoperative blood loss, preventing the occurrence of bladder perforation, and also reducing the obstacles of electrocoagulation hemostasis, so that hemostasis is more sufficient, which helps to shorten the postoperative hospital stay of patients [23]. In addition, when bladder tumor resection is performed, because the surgeon is excessively worried about the occurrence of obturator nerve reflex, it may lead to incomplete tumor resection, which leads to tumor recurrence, while obturator nerve block can reduce tumor recurrence [24].

In the literature [16], the study compared the changes of serum TNF-*α*, IL-6, and IL-8 levels between the two groups after TURBT surgery, and the results showed that the serum TNF-*α*, IL-6, and IL-8 levels were increased in both groups after surgery, but the observation group was lower than the control group, which indicated that SA combined with ONB could reduce the trauma during surgery, reduce the inflammatory stress response, and facilitate postoperative recovery. However, because only serum inflammatory parameters have been reported in the literature [16], we did not conduct a pooled analysis of this indicator.

Although there was no heterogeneity in the literature studies in the analysis process, we still performed a subgroup analysis, and the transinguinal approach showed a significant difference from the transphobic approach. In obturator nerve block, the pubic puncture approach has disadvantages such as large needle insertion depth and a large dose of anesthetic drugs, on the contrary, the inguinal approach has advantages such as superficial needle insertion and mild puncture pain [25], therefore, the safety of the transinguinal approach is better, but the comparison of the two approaches still needs to be confirmed by more clinical controlled studies.

Among the 8 literature studies included in this study, 2 literature studies used ultrasound-guided nerve stimulation while the other 6 literature studies used nerve electrical stimulation. A meta-analysis study [26] concluded that both techniques were safe in the implementation of ONB. However, using nerve stimulation as an auxiliary means would be more accurate in the localization, faster in the onset of block, and higher in the success rate.

This study still has some limitations, which are reflected in: ①the number of included literature studies is small, the number of patients participating is still small, and there is a lack of multicenter, large-sample size randomized controlled trials; ②some literature studies do not describe the allocation concealment, do not describe the blind method, do not count the dropout cases, and there may be certain bias; and ③the effectiveness of ONB is affected by a variety of factors, such as puncture approach, ultrasound technology, the use of anesthetic drug dose, and the selection of current intensity, but there are too few included studies to compare a variety of groups.

## 5. Conclusion

In summary, the application of spinal anesthesia combined with obturator nerve block in TURBT surgery can effectively reduce the incidence of obturator nerve reflex, reduce the incidence of bladder perforation, shorten the hospital stay, and reduce the tumor recurrence rate, but more high-quality, multicenter, large-sample randomized controlled studies need to be included in clinical practice to provide stronger evidence.

## Figures and Tables

**Figure 1:** Literature selection flow chart.

**Figure 2:** Comparison of the incidence of bladder perforation between SA + ONB and SA alone in TURBT.

**Figure 3:** Comparison of the incidence of obturator nerve reflex between SA + ONB and SA alone in TURBT.

**Figure 4:** Comparison of hospital stay after TURBT between SA + ONB and SA alone.

**Figure 5:** Comparison of tumor recurrence rate after TURBT between SA + ONB and SA alone.

**Figure 6:** Sensitivity analysis of incidence indicators of bladder perforation.

**Figure 7:** Funnel plot analysis of incidence indicators of bladder perforation.

**Table 1:** Basic characteristics, intervention measures, outcome indicators, and quality scores of the included literature.

Author	Year	Mean age (years)	Spinal anesthesia method	ONB anesthetic drugs and dose	Approach	Ultrasound guidance/nerve stimulator	Population (*E*/*C*)	Follow-up time (mo)	Outcome indicators	Jadad score
Doluoglu et al. [10]	2021	64.6 ± 11.7	Spinal block	1% lidocaine 10 mL	Inguen	Neurostimulation	61/62	32.3 ± 5.3	①②④⑤	4

Tekül et al. [11]	2014	65.8 ± 7.8	Spinal block	0.25% levobupivacaine 10 mL	The pubic tubercle	Neurostimulation	32/36	31.6 ± 5.9	⑤	4

Bolat et al. [12]	2015	67.7 ± 10.5	Spinal block	0.25% levobupivacaine 10 mL	The pubic tubercle	Neurostimulation	35/35	N/A	①②	4

Khorrami et al. [13]	2010	62 ± 11	Spinal block	1% lidocaine 10 mL	Inguen	Neurostimulation	30/30	N/A	⑦	4

Erbay et al. [14]	2017	69.2 (31–89)	Spinal block	1% lidocaine 10 mL	Inguen	Neurostimulation	47/49	36.3 ± 17.2	①②⑤⑥	3

Alavi et al. [15]	2017	67 (50–79)	Spinal block	1% lidocaine 10 mL	The pubic tubercle	Neurostimulation	15/15	N/A	②	4

Yu et al. [16]	2021	61.45 ± 10.36	Spinal epidural	0.5% lidocaine 10 mL	Inguen	Ultrasound guidance	45/45	N/A	①②③④	2

Wu et al. [17]	2016	62.9 (28–84)	Spinal epidural	1% lidocaine 10 mL	Inguen	Ultrasound guidance	50/48	20.71 ± 12.32	①③④⑤	2

E: intervention group, C: control group; N/A: not available; ONB: Obturator nerve block. Outcomes: ①incidence of bladder perforation; ②incidence of obturator reflex; ③indwelling time of urinary catheter; ④length of hospital stay; ⑤tumor recurrence rate during follow-up; ⑥survival rate.

**Table 2:** Risk of bias based on the cochrane handbook for evaluation of randomized interventions.

Study	Random sequence generation	Classification hiding	Blind method	Data integrity	Optional reporting	Other bias
Doluoglu et al. [10]	Low	Low	Low	Low	Low	Low
Tekül et al. [11]	Low	Low	Low	Low	Low	Low
Bolat et al. [12]	Low	Low	Low	Low	Low	Low
Khorrami et al. [13]	Low	Low	Low	Low	Low	Low
Erbay et al. [14]	Low	Unclear	Low	Low	Low	Low
Alavi et al. [15]	Low	Low	Low	Low	Low	Low
Yu et al. [16]	Low	Unclear	Unclear	Unclear	Low	Low
Wu et al. [17]	Low	Unclear	Unclear	Unclear	Low	Low

## Data Availability

The data can be obtained from the author upon reasonable request.
